This article has been retracted.

# Facile Synthesis of NaYF4:Yb Up-Conversion Nanoparticles Modified with Photosensitizer and Targeting Antibody for In Vitro Photodynamic Therapy of Hepatocellular Carcinoma

**DOI:** 10.1155/2022/4470510

**Published:** 2022-03-08

**Authors:** Jingyi Ding, Yan Jin, Fengqi Zhu, Cunle Zhu, Jiang Peng, Tiantian Su, Jinzhen Cai

**Affiliations:** ^1^The Institute of Transplantation Science, Qingdao University, Qingdao 266000, China; ^2^Department of Human Anatomy, Histology and Embryology, Key Laboratory of Carcinogenesis and Translational Research (Ministry of Education) and State Key Laboratory of Natural and Biomimetic Drugs, Peking University Health Science Center, Beijing 100086, China; ^3^Organ Transplantation Center, The Institute of Transplantation Science, The Affiliated Hospital of Qingdao University, Qingdao 266000, China

## Abstract

Rare Earth up-conversion nanoparticles NaYF4:20%Yb,2%Er@PEI (UCNPs) were generated via a one-step hydrothermal technique at relatively reduced temperatures. Photosensitizer Ce6 and anti-EpCAM, a highly expressed monoclonal antibody in cancer stem cells of hepatocellular carcinoma, were linked to UCNP surfaces via the formation of amide linkage between carboxyl from Ce6 or anti-EpCAM and abundant amino from PEI, leading to the formation of Ps-Ce6 and anti-EpCAM-UCNPs-Ce6 nanoparticles. The synthesized nanoparticles characterized by XRD, TEM, and IR, and their zeta potential, ROS generation ability, Ce6 loading rate, and up-conversion fluorescence properties were investigated. It has been revealed that all the products were uniformly dispersed nanoparticles (25–32 nm), which crystallized primarily as hexagonal structures, and their up-conversion fluorescence spectra were similar to that of NaYF4:20%Yb,2%Er. The Ce6 loading rate in the anti-EpCAM-UCNPs-Ce6 nanoparticles was about 2.9%, thereby resulting in good ROS generation ability. For anti-EpCAM-UCNPs-Ce6, the biosafety, targeting effect, and PDT effect exposed under near-infrared (NIR) laser (980 nm) were evaluated using human liver cancer cells (BEL-7404). The results showed that it has good biocompatibility and biosafety as well as high targeting and PDT treatment efficiencies, which renders it a potential experimental material for the near-infrared PDT study.

## 1. Introduction

As one of the most common malignant tumors globally, morbidity and mortality rates for hepatic tumors rank 6th and 4th, respectively, from all clinically observed tumor models [1]. Due to the insidious condition progression, it is typically not detected until such an illness is in the middle or advanced stages, and the 5-year survival rate is as low as 10.1%, accompanied by a poor life quality of patients [2]. Currently, chemotherapy, radiotherapy, immunotherapy, and arterial chemoembolization are the major available options for treating middle-advanced liver cancer [3]. However, there are quite a few disadvantages of these methods, such as systemic toxicity, radiation damage, low selectivity as well as drug resistance [4, 5]; hence, developing safe and efficient treatment plans for malignant tumors is a major need.

Recently, nanomaterial-based photodynamic therapy (PDT) has received wide attention and has become an important research niche for cancer treatment [6, 7]. PDT is a noninvasive treatment, and its basic principle is as follows: after the photosensitizer ingested by the tumor cells is excited by light of a certain wavelength, it is capable of transferring the absorbed energy to the ambient oxygen present, developing reactive oxygen species (ROS) that can lead to oxidation-driven dysfunction within mitochondria and DNA, causing cell apoptosis and necrosis, thereby curing cancer [8]. In comparison to traditional cancer treatments, PDT has several advantages, such as less trauma, good applicability, accurate targeting, low toxicity, and low cost, and is well established in treating esophageal tumors, skin cancer, and other tumors with excellent curative effect [9–11]. However, most photosensitizers used in traditional PDT treatment are porphyrins or phthalocyanine derivatives, which suffer from poor hydrophilicity and biocompatibility, and cannot be easily transported to the tumor site [12, 13]. Furthermore, the ultraviolet-visible (UV-Vis) light for exciting the photosensitizer is easily absorbed or quenched by biological tissues, thus the depth of penetration is minimized, and it can easily cause light damage to biological tissues. Therefore, PDT treatment is now limited to the treatment of superficial or tiny tumors, but the impact of the treatment of traditional PDT for deep tumors is rather unsatisfactory [14, 15].

Up-conversion luminescent materials can convert long-wave radiation with lower energy to short-wave radiation with higher energy mediated by two-/multi-photon techniques, also referred to as antiStokes shift [16]. For example, hexagonal*β*-NaYF4:Yb, Er is a well-known up-conversion luminescent material with high efficiency, which can generate UV-Vis fluorescence with high intensity and low-nonspecific fluorescence background under the excitation of near-infrared (NIR) laser [17]. More importantly, the infrared band (700–1000 nm) lies inside a bio-optical window, which can reduce the extent of light absorption by biological tissues. In addition, the penetrability of NIR into tissue is stronger, and the light damage of NIR to the organism is relatively less in comparison to that of ultraviolet light [18]. The up-conversion nanoparticles (UCNPs) suitable for biological application can be synthesized with many chemical methods together with further surface functional modification by photosensitizers, hydrophilic groups, targeting agent, specific antibodies, and so on, to facilitate the PDT for deep-tissue cancers, improving selectivity and biocompatibility and reducing side effects [19–21].

The materials used in PDT must be very small monodisperse nanoparticles having good water solubility. Monodisperse *β*-NaYF4:Yb, Er nanoparticles, having a high intensity of up-conversion fluorescence, were usually synthesized through pyrolysis method comprising dissolution, precursor formation (150°C), distillation for the removal of methanol (70°C), and pyrolysis (300–320°C) for promoting the cubic-to-hexagonal phase transformation [22]. However, there are some obvious disadvantages of this method, such as complicated and long procedure, production of large amount refractory waste solvent due to the oxidation, polymerization, and pyrolysis of octadecene and oleic acid upon attaining elevated temperatures. Furthermore, the oleic acid linked to *β*-NaYF4:Yb, Er surfaces is highly hydrophobic; thus, it needs to be removed and subsequently substituted by hydrophilic groups through various kinds of physical and chemical methods.

Polyethyleneimine (PEI) has a large number of amino groups with high reactivity and polarity and an abundance of positive charges. Accordingly, surface modification of the *β*-NaYF4:Yb, Er nanoparticles by PEI could not only increase the hydrophilicity but also conveniently increment the reactive activity for further functionalization. At the same time, the positive charge on the PEI surface can adhere to negatively charged residues upon cellular surfaces and penetrate via endocytosis for promoting drug uptake, a phenomenon known as enhanced permeability and retention effect (EPR) [23, 24].

However, relying only on the EPR causes passive accumulation of UCNP in the body, reducing the overall therapeutic effect. If some specific molecules are conjugated onto the surface of UCNPs, such as the monoclonal antibody anti-EpCAM, which can target the surface marker epithelial cell adhesion molecule (EpCAM) of the cancer stem cells of hepatocellular carcinoma, the nanosystem would possess an active targeting effect. EpCAM consists of a transmembrane glycoprotein that is mainly present within epithelial/progenitor/normal/malignant stem cells and a variety of tumor cells [25]. EpCAM expression profile changes dynamically throughout hepatic maturation. It can be detected in both bile duct plate cells and liver parenchyma cells within fetal/neonatal livers, particularly in the former, then decreases significantly with age till it practically disappears in the liver of healthy adults [26, 27]. However, during the occurrence and development of hepatocellular carcinoma, liver pathological changes are linked to potent EpCAM reexpression, and EpCAM expression by liver cancer cells is significantly higher in comparison to that in normal epithelial cells [28]. If the anti-EpCAM and photosensitizer are assembled on the surface of UCNPs via chemical reactions, it would presumably result in a good NIR-PDT method with high targeting ability and low side effects for hepatocellular carcinoma. There are a few reports on the conjugation of specific antibodies with UCNPs; however, most of them were coated with mesoporous silica. Surface modification of UCNPs with both specific antibodies and photosensitizer by using PEI as a bridge has been rarely reported [29, 30].

In this study, monodisperse UCNPs (*β*-NaYF4:Yb, Er@PEI) were generated via one-step hydrothermal technique at a relatively reduced temperature. The photosensitizer chlorin e6 (Ce6) and anti-EpCAM were further assembled over UCNP surfaces through the formation of amide linkage, constructing an anti-EpCAM-UCNPs-Ce6 nanoplatform, which was identified through X-ray diffraction (XRD), transmission electron microscopy (TEM), infrared spectrum (IR), and UV-Vis spectrum. In addition, the cell line BEL7404 was used to evaluate the biosafety of anti-EpCAM-UCNPs-Ce6, and in-cell PDT and cell-targeted uptake experiments were conducted to provide basic data for the clinical application of the system. The principle of PDT for liver cancer cells based on upconversion nanoparticles modified by Ce6 and anti-EpCAM is shown in Scheme 1.

## 2. Methodology

### 2.1. Materials and Cell Lines

Er(NO_3_)_3_·5H_2_O (99.9%), Yb(NO_3_)_3_·5H_2_O (99.9%), Y(NO_3_)_3_·6H_2_O (99.9%), NaOH (analytical purity AR), absolute ethanol (AR), hydroxyethyl cellulose (AR, viscosity of 20,000 mPa s), polyethyleneimine (PEI, M.W. = 10000, 99%), NH4F (98%), concentrated hydrochloric acid (AR, 37%), dimethyl sulfoxide (DMSO, AR), 1-(3-dimethylamino propyl)-3-ethyl-carbodiimide hydrochloride (EDC, 98%), N-hydroxysuccinimide (NHS, 98%), phosphate-buffered saline (PBS, pH = 7.2–7.4), chlorin E6 (Ce6, 94%), and 1,3-diphenylisobenzofuran (DPBF, 99.9%) were procured through Sigma-Aldrich™ (St. Louis, USA). Anti-EpCAM monoclonal antibody was procured through eBioscience (San Diego, USA). A cellular proliferation kit (CCK-8) was procured through Abcam™ (Shanghai, China). 4′,6-Diamidino-2-phenylindole, dihydrochloride (DAPI) was procured through Sigma-Aldrich Chemicals™ (Sydney, Australia).

The human hepatocellular carcinoma cell line BEL-7404 was obtained from ATCC (Shanghai, China), and the LO_2_ cell line was obtained from the Affiliated Hospital of Qingdao University, China. BEL-7404 cultures were grown within RPMI-1640 medium, and LO_2_ cells were grown within DMEM augmented by 10% fetal bovine serum (FBS)/1% penicillin-streptomycin at 37°C within a humidified atmosphere carrying 5% CO_2_.

### 2.2. Generation of Targeted UCNPs

#### 2.2.1. Generation of NaYF4:20%Yb,2%Er@PEI (UCNPs)

For creating UCNPs, 0.5 g NaOH, 0.5 g YCl_3_.7H_2_O (1.56 mmol), 0.15 g YbCl_3_.6H_2_O (0.4 mmol), 0.015 g ErCl_3_.6H_2_O (0.04 mmol), 1.0 g polyethylene imine (PEI, AR, *M* = 20,000), 0.5 g NH_4_F, 0.2 g hydroxyethyl cellulose (AR, viscosity of 20,000 mpa s), and 40 ml deionized water were added to the inner tank of a polytetrafluoroethylene reactor and stirred evenly to yield a viscous semifluid. The pH was optimized for 6.5–7.0 using 6 M HCl, and then the stainless reactor shell was applied to seal the reactor. The reactor was placed in a homogeneous reactor with a rotating shaft at 80 rpm, allowed to react at 150°C for 10 hours, and left to cool down naturally after the reaction. The initial product was centrifuged at 5,000 rpm (5 minutes), mother liquor was removed, with the precipitate washed three times using 5 mL deionized water (5,000 rpm). Subsequently, 5 ml DMSO was added to the washed precipitate for ultrasonic dispersion and centrifuged at 14,000 rpm, and the mother liquor was discarded. The precipitate was centrifuged again and washed with DMSO thrice, and the solid products were freeze dried.

#### 2.2.2. Synthesis of UCNPs-Ce6

The activated Ce6 solution was obtained by dispersing 5 mg Ce6, 15 mg EDC, and 15 mg NHS within 25 mL DMSO, with the solution mixed at ambient temperature for 120 minutes. Consequently, 20 mg UCNPs were added into 10 mL DMSO and dispersed by ultrasonication to obtain a uniform solution. The solution was mixed with the activated Ce6 solution, stirred at room temperature, and reacted in dark for 12 hours. After the reaction, the product was centrifuged (14,000 rpm), and the mother liquor was removed, with crude solid product washed using 5 mL DMSO thrice and subsequently freeze dried.

#### 2.2.3. Synthesis of Anti-EpCAM-UCNPs-Ce6

The mixture of UCNPs-Ce6 (2 mg) and PBS buffer (10 ml) was shaken for 30 minutes, centrifuged, with precipitate washed four times using PBS (14,000 rpm). Then 10 mL PBS and 40 *μ*g anti-EpCAM were introduced into obtained solid, and the mixture was shaken completely (30 minutes) and then centrifuged. Precipitate was washed thrice using PBS for removing unreacted antibodies, with such product being ultrasonically dispersed in PBS. The schematic diagram of the material synthesis is shown in Figures 1 and 2.

### 2.3. Characterization of Nanomaterials

An X-ray diffractometer was used to record the XRD patterns to characterize the phase of the materials, using Cu K*α* (*λ* = 1.54056 Å) as the radiation source at a functional voltage of 40 kV, a functional current of 100 mA, a scanning rate of 8°/min, and a step size of 0.02°.

IR spectrums of the materials were recorded using the potassium bromide pressed-disk method to detect the characteristic functional groups across material surfaces. Scanning range was 650–4000 cm^−1^, and the resolution was 4 cm^−1^.

TEM images were taken by JEM-2100F TEM in bright-field mode at an operating voltage of 200 kV to determine the morphology and size of the materials. The sample preparation for TEM microscopy is as follows: the freeze-dried materials were dispersed in ethanol solution at a concentration of about 0.1 mg/mL, which were ultrasonicated for 10 minutes. Then, 10 *μ*L of the solution was dropped onto the carbon film microgrid and dried naturally.

The nanoparticles were ultrasonically dispersed in deionized water for 15 minutes to record the fluorescence spectrums by using a fluorescence spectrophotometer with a 980 nm laser (IR range) as an excitation source. Test condition is as follows: 1 kW of the power of the laser, 0.2 nm of the emission slit, and 450–700 nm of the scanning range.

The zeta potentials of the nanoparticles, which were dispersed into de-ionized water to render a solution (2 mg/mL), were measured with a zeta potentiometer (SOE-070) at 25°C.

### 2.4. ROS Generation Ability Detection

After DPBF captured the ROS generated by the photosensitizer, the absorption intensity between 350 and 470 nm weakened. UCNPs-Ce6 was dispersed in DPBF-ethanol as a solution of 50 mg/L standing in the dark for 1 hour allowing DPBF to adsorb UCNPs-Ce6. The solution was irradiated using a 980 nm laser (power density = 1.0 W/cm^2^) and sampled every 5 minutes. UV-Vis absorption spectra for this solution were determined using UV-Vis spectrophotometry. Test conditions were as follows: scanning range: 200 nm–1100 nm; slit width: 2.0 nm, and sampling interval: 0.5 nm. The absorption peak intensity-time curve was drawn at 420 nm.

## 3. Cellular Experiments

### 3.1. Nanoparticle Cytotoxicity Test

As a potential material for use in human therapy, the nanoparticles must have low toxicity. Normal human liver cells (LO_2_) were employed for evaluating in vitro cytotoxicity by synthesized nanoparticles. LO_2_ cultures were introduced into a 96-well plate (2 × 103 cells/well) and placed into incubation at 37°C and 5% CO_2_ (approximately 12 hours). The UCNPs/UCNPs-Ce6/anti-EpCAM-UCNPs-Ce6 were divided into two groups, cultured with DMEM medium, and used to prepare solutions at different concentrations (3.9–500 *μ*g/mL). Each group was tested in three wells, along with the blank control group, and cultured at 37°C and 5% CO_2_ (24 and 48 h, respectively). Experimental cultures and 100 *μ*L CCK-8 were incubated for 4 hours. Optical density value (OD value) for individual wells was calculated through a microplate reader at 450 nm, using the following formula for cellular inhibition rates: inhibition rate = ((OD value of control group − OD value of treatment group)/OD value of control group) × 100%.

### 3.2. Targeting Uptake Ability of Anti-EpCAM-UCNPs-Ce6

In order to probe the targeting ability for generated nanoparticles, we used human liver cancer cell line BEL-7404 (2 × 103 cells/well), in which the EpCAM expression rate as measured by flow cytometry was 51.55%. The BEL-7404 cells (2 × 103 cells/well) were inoculated into 6-well plates until the adherent growth reached about 80%. The cells were exposed to 200 *μ*g/mL anti-EpCAM-UCNPs together with nontargeted UCNPs (not combined with anti-EpCAM) and pretreated with 20 *μ*L of free anti-EpCAM (0.1 *μ*g/mL) for the blocking test. In the next step, cultures were washed thrice using PBS for removing free nanoparticles. Cultures were placed again into incubation with 2 *μ*g/mL DAPI for nuclear staining. Then, samples were observed and detected using an external 980 nm light source under an inverted fluorescence microscope. Image J software was employed for semiquantitative calculation of the green fluorescence intensity of the cytoplasm in each group.

### 3.3. Effect of External PDT of Anti-EpCAM-UCNPs-Ce6

Bel-7404 cells were plated into 6-well plates (105 cells/well) and cultured at 37°C and 5% CO_2_ for 24 hours. Cultures were divided into a NIR group, Ce6 group, UCNPs-Ce6 group, anti-EpCAM-UCNPs-Ce6 group, and UCNPs group. An RPMI1640 (medium) group served as control group. The concentration gradient for Ce6 was 1 *μ*g/mL. Cultures were irradiated through a 980 nm NIR laser (power density = 320 mW/cm^2^ for 5 minutes) and then placed in a cell incubator for further culturing for 24 hours. The survival rate of the cells was determined (450 nm) in a microplate reader. The CCK-8 was used to measure cellular proliferation in this experiment.

## 4. Results and Discussion

### 4.1. Phase and Morphology Analysis

The XRD patterns of UCNPs and UCNPs-Ce6 are shown in Figure 3. The results show that the two exist in similar phases, indicating that the crystal structure of the UCNPs did not change following the attachment of Ce6 to the surface. The main phase was isomorphic to hexagonal NaYF4 (*β*-NaYF4, JCPDS 16-0344), and some were isomorphic to cubic NaYF4 (*β*-NaYF4, JCPDS 77-2042), with a small amount of unknown impurities.

Figures 4(a)–4(c) are TEM photos of UCNPs, UCNPs-Ce6, and anti-EpCAM-UCNPs-Ce6. Their particle sizes are approximately 25 nm, 28 nm, and 32 nm, respectively. All nanoparticles had good dispersibility and are suitable for biological applications.

UCNPs nanoparticles that mainly crystallized in a hexagonal structure, in this study, were generated using one-step hydrothermal technique through hydroxyethyl cellulose serving as a crystal growth inhibitorandPEI as a surface modifier. The products had a high polarity and good water dispersion properties. The reaction temperature (150°C) for this method was significantly lower than that used in the high-temperature thermal decomposition method [22]. Besides, the synthesis step was simple, without employing any long-chain fatty acids, thereby avoiding the complicated postprocessing process, which thus opens new paths for the research and application of *β*-NaYF_4_-based up-conversion fluorescent materials.

### 4.2. IR and Zeta Potential Analysis

Figure 5 shows the IR spectra for UCNPs, UCNPs-Ce6, and anti-EpCAM-UCNPs-Ce6. Regarding IR spectrum for UCNPs, the peaks occurring at 3427, 2957, 1470, and 1314 cm^−1^ correspond to N-H stretching vibrations, C-H stretching/bending vibrations, and C-N stretching vibrations, respectively, which all originated from PEI, indicating that PEI successfully modified NaYF4:20%Yb, 2%Er nanoparticle surfaces, and abundant amino groups increased the polarity of the UCNPs, resulting in good hydrophilicity. On the other hand, no C-O stretching vibration peaks (strong and wide peak between 1000 and 1200 cm^−1^) were observed, indicating that hydroxyethyl cellulose is only used as a reaction medium during the synthesis process, whose role was to probably form a uniform dense gel inhibiting the growth of UCNPs particles.

Regarding IR spectrum for UCNPs-Ce6, peaks appearing at 3422, 2967, 1652, 1541, 1455, 1267, and 1116 cm^−1^ corresponded to N-H and O-H and/or C-H stretching vibrations, C=O stretching vibrations, N-H bending vibrations in amide, C-H stretching vibrations, C-N stretching vibrations, and C-O stretching vibrations, respectively. Besides absorption peaks for characteristic PEI groups, there were also characteristic peaks for C=O, C-O, and amide N-H bending vibrations, which indicated that amide bond formation reaction occurred between -NH2 from PEI on the surface of UCNPs and -COOH from Ce6; thereupon, then the photosensitizer Ce6 was firmly and chemically bonded to the surface of the upconversion nanomaterial. However, the conjugate structure of Ce6 itself did not change, thus it still could generate ROS under the excitation of visible light at a certain wavelength and can be used as the active component of PDT.

In the IR spectrum of anti-EpCAM-UCNPs-Ce6 the peaks at 3357, 2936, 1642, 1557, 1445, 1267, 1197, 1121, 909 cm^−1^ were in line with N-H stretching vibrations and O-H stretching vibrations, C-H stretching vibrations, C=O stretching vibrations in amide, N-H bending vibrations in amide, C-H stretching vibrations, C-N stretching vibrations, P=O stretching vibrations, C-O stretching vibrations, and P-O-C stretching vibrations. In addition to the IR absorption peaks of the characteristic groups of UCNPs-Ce6, there were also P=O stretching vibrations and P-O-C stretching vibrations, which came from the phospholipid acyl group in the anti-EpCAM antibody, indicating that anti-EpCAM was successfully loaded onto the surface of the nanoparticles.

UCNPs, UCNPs-Ce6, and anti-EpCAM-UCNPs-Ce6 had zeta potentials of 32.1, 17.5, and 10.2 mV, respectively. Due to the abundance of positive charges on the surface of PEI, UCNPs treated simply with PEI have a rather high zeta potential. The zeta potentials of Ce6 and anti-EpCAM were reduced to 17.5 mV and 10.2 mV, respectively, when they chemically bound to the amino groups on the PEI surface, substantially reducing the damage caused by positive charges on cell membranes. The modest amount of positive charge on the surface of nanoparticles, on the other hand, prevents nanoparticle aggregation and allows them to penetrate cells.

### 4.3. ROS Generation Ability

DPBF is a commonly used ROS-capture agent. After it is oxidized by ROS, the characteristic absorption peak in the 350∼450 nm range would be significantly weakened. Therefore, DPBF can be used to detect the ability of materials to generate ROS. To 5 mL of anti-EpCAM-UCNPs-Ce6 ethanol solution (2 mg/mL), 0.5 mg DPBF were introduced, with such mixture stirred in dark conditions. The mixed solution was simultaneously irradiated with a 980 nm laser (1.0 W/cm^2^) for various timeframes. Postirradiation, the mixture solution was centrifugated at 13,000 rpm for 5 minutes to discard the anti-EpCAM-UCNPs-Ce6 nanoparticles, with UV-Vis spectra of the supernatant determined.  Figure 6 shows the UV-Vis spectra of eight samples subjected to the same treatment process and irradiation for 0, 5, 10, 15, 20, 25, and 35 minutes, respectively. The results show that, with the prolongation of irradiation time, the intensity of the characteristic absorption peaks in the 350∼450 nm range gradually decreased, indicating that anti-EpCAM-UCNPs-Ce6 generated ROS under 980 nm infrared laser irradiation, which demonstrates its potential for application in PDT research fields.

### 4.4. Ce6 Loading Rate Testing

A predetermined amount of Ce6 was dissolved in ethanol to form a series of solutions of 1, 5, 10, 15, and 20 *μ*g/mL. The absorbance of these solutions at the maximum absorption wavelength of Ce6 (404 nm) was determined through UV-Vis spectrophotometry, and the standard curve of Ce6 absorbance against concentration was drawn, as shown in Figure 7. The linear regression equation for the standard curve was *A* = 0.216*c* − 0.001, and the correlation coefficient was *R* = 0.9929. Then, 2 mg anti-EpCAM-UCNPs-Ce6 was added to 5 mL ethanol and dispersed uniformly via ultrasonication to form the solution of nanoparticles, and its absorbance at 404 nm was determined through UV-Vis spectrophotometry. According to such calculation, [Ce6] in anti-EpCAM-UCNPs-Ce6 was 11.56 (*μ*g/mL) × 5 mL/2 mg = 2.9%.

### 4.5. Up-Conversion Fluorescence Properties

The nanoparticles were dispersed in deionized water and homogenized ultrasonically for 15 minutes to produce an aqueous nanoparticle dispersion of 1 mg/mL to record their up-conversion fluorescence spectrum under the excitation of a 980 nm infrared laser having 1.0 kW power. As shown in Figure 8, the emission spectra for UCNPs, UCNPs-Ce6, and anti-EpCAM-UCNPs-Ce6 were quite similar to the up-conversion fluorescence spectra of NaYF4:20%Yb,2%Er reported in many previous reports [17, 22], which indicates that the surface modifications of UCNPs by Ce6 and anti-EpCAM do not change their up-conversion fluorescence properties but decrease the fluorescence intensity of the materials. Ce6 can produce ROS under the excitation of the up-conversion fluorescence, which demonstrates their potential for use in PDT.

### 4.6. Nanomaterial Toxicity Tests

The cytotoxicity of the UCNPs, UCNPs-Ce6, and anti-EpCAM-UCNPs-Ce6 nanoparticles on human normal hepatocytes (LO_2_) was demonstrated by CCK-8 testing. PEI has a large amount of positive charge on its surface, which is destructive to cell membranes and has a demonstrated cytotoxicity. However, as evident from Figure 9, UCNPs have low toxicity, which is presumably because the protonated amino nitrogen atoms on the PEI surface replace some of the Na+ in *β*-NaYF4:Yb, Er, thus reducing the number of surface positive charges. With the surface modification of UCNPs by Ce6 and anti-EpCAM, the positive charge on the surface of the entire nanoparticle is further reduced. This observation is also quite consistent with the zeta potential values (32.1, 17.5, and 10.2 mV) recorded for the above three materials. The PEI coated on the surface of anti-EpCAM-UCNPs-Ce6 material contains an abundance of polar groups, which confers increased water solubility. Meanwhile, the coupling of the photosensitizer and specific antibody with amino groups on the surface of PEI not only introduces photoactive and targeting groups but also significantly reduces its cytotoxicity, thus rendering good biocompatibility. The cell survival rate was highest when anti-EpCAM-UCNPs-Ce6 was applied at the highest concentration (500 *μ*g/mL).

### 4.7. In Vitro Targeting Ability of the Nanomaterial

The anti-EpCAM monoclonal antibody was used to label the BEL-7404 cell line. The flow cytometric analysis revealed that the EpCAM expression rate of this cell line was 51.5%, as shown in Figure 10. Inverted fluorescence was employed for monitoring potential by anti-Epti-EpCAM-UCNPs to target the EpCAM-positive hepatoma cell BEL-7404. As seen in Figure 10, the targeted group's cytoplasm had a strong green, fluorescent signal, indicating that the EpCAM antibody conjugated to the targeted material group had interacted with the EpCAM antigen on the cell surface, enhancing the cells' absorption capacity for the materials. However, there was a small amount of fluorescent signal in the cytoplasm of the nontargeted group, which could be because the nontargeted material only entered the cells through nonspecific endocytosis. This implies that its intake was markedly reduced in comparison to targeted material. Cultures in the blocking group were first treated with an anti-EpCAM monoclonal antibody for 4 hours before being incubated with anti-EpCAM-UCNPs. After washing, the intensity of the green, fluorescent signal in the cytoplasm was the lowest among the three groups. This is because, after pretreatment with an anti-EpCAM monoclonal antibody, the antigen-binding site on the cell was blocked, resulting in a significant reduction in the uptake of targeted nanomaterials by the cell and a weak green signal. The semiquantitative analysis of the green fluorescence signal of each group by Image J showed that the results were consistent with the observations under an inverted fluorescence microscope, and the fluorescent signal values of each group were significantly different statistically. The results showed that the EpCAM antibody ligand enhanced the uptake of nanoparticles by hepatocellular carcinoma cells.

### 4.8. In Vitro Antitumor Effect Study

To test the antitumor influence by nanoparticles when excited at 980 nm NIR light in vitro, a 980 nm NIR laser (power density of 320 mW/cm^2^) was used to irradiate the material, and cells in the NIR group, control group (RMPI1640), Ce6 (100 *μ*g, concentration: 1 *μ*g/ml), Ce6-UCNPs group (100 *μ*g), anti-EpCAM-UCNPs-Ce6 group (100 *μ*g), and UCNPs (100 *μ*g) group were analyzed with the CCK-8. As shown in Figure 11, 980 nm NIR irradiation alone had no significant cell-killing ability, the cell death rate in the anti-EpCAM-UCNPs-Ce6 group was markedly elevated in comparison to other groups, and the apoptotic rate was 87.57% for 100 *μ*g/mL anti-EpCAM-UCNPs-Ce6.

## 5. Conclusion

In this research, an up-conversion nanoplatform (anti-EpCAM-UCNPs-Ce6) comodified by Ce6 and anti-EpCAM was successfully fabricated. The preparation process avoided the traditional high-temperature pyrolysis as well as solvent wastage This platform organically combines the effects of NIR PDT—low light damage and deep tissue penetration—with the targeting properties of anti-EpCAM and shows good biocompatibility and excellent up-conversion fluorescence performance. In vitro experiments showed that the platform has good biosafety, targeting, and PDT tumor treatment effects under the action of NIR light (980 nm).

## Figures and Tables

**Scheme 1:** Schematic diagram depicting PDT therapy of anti-EpCAM-UCNPs-Ce6 nanoplatform in vivo. After binding with EpCAM-expressing hepatoma cells, PDT could be achieved after irradiation at 980 nm.

**Figure 1:** Schematic diagram illustrating the hydrothermal generation of NaYF4:20%Yb,2%Er@PEI(UCNPs).

**Figure 2:** Schematic diagram illustrating UCNPs surface modification.

**Figure 3:** XRD patterns of UCNPs and UCNPs-Ce6 nanoparticle powders, in which *H* is the diffraction peak for hexagonal phase, *C* is the diffraction peak for cubic phase, and *X* is the diffraction peak of unknown impurities.

**Figure 4:** TEM images of powdered nanoparticles. (a) UCNPs. (b) UCNPs-Ce6. (c) Anti-EpCAM-UCNPs-Ce6.

**Figure 5:** IR spectra of UCNPs, UCNPs-Ce6, and anti-EpCAM-UCNPs-Ce6.

**Figure 6:** Anti-EpCAM-UCNPs-Ce6 after being adsorbed, the variation of the characteristic absorption peak of the ultraviolet spectrum (350–450 nm) of DPBF with the irradiation time of infrared laser (980 nm).

**Figure 7:** Standard curve and the load rate of Ce6.

**Figure 8:** Up-conversion fluorescence spectra for UCNPs, UCNPs-Ce6, and anti-EpCAM-UCNPs-Ce6 under the excitation of 980 nm infrared laser.

**Figure 9:** Cytotoxicity assay results of the anti-EpCAM-UCNPs-Ce6 nanoplatform. (a) Cell viability of LO_2_ cells following 24 h coincubation with different concentrations of anti-EpCAM-UCNPs-Ce6/UCNPs/UCNPs-Ce6. (b) Cell viability of LO_2_ cells incubated with differing doses of anti-EpCAM-UCNPs-Ce6/UCNPs/UCNPs-Ce6 for 48 h.

**Figure 10:** Results of in vitro targeting of materials evaluated by fluorescence inversion. (a) Results of UCNPs-ce6 coincubation with BEL-7404 cells after 4 h. (b) Results of BEL-7404 cells photographed after 4 h incubation with anti-EpCAM-UCNPs-ce6. (c) The result after coincubation of BEL-7404 cells with an anti-EpCAM monoclonal antibody, followed by coincubation with anti-EpCAM-UCNPs-ce6 for 4 h. (d) Semiquantitative plots of cellular fluorescence values in different treatment groups (^*∗∗∗∗*^*P* < 0.0001). EpCAM expression in the BEL-7404 cell line. (e) Flow cytometric plot of cells and anti-EpCAM monoclonal antibody after coculture. (f) Blank control: graph of the flow results of cells without any labeling.

**Figure 11:** Results of the PDT effect study of the anti-EpCAM-UCNPs-Ce6 nanoplatform. The figure shows the survival of BEL-7404 after being given different conditions.

## Data Availability

The data that support the findings of this study are available from the corresponding author upon reasonable request.

## Abbreviations

UCNPs: Up-conversion nanoparticles
PDT: Photodynamic therapy
PEI: Polyethyleneimine
Ce6: Chlorin e6
Anti-EpCAM: Epithelial cell adhesion molecule antibody
XRD: X-ray diffraction
TEM: Transmission electron microscope
IR: Infrared spectrum
ROS: Reactive oxygen species
NIR: Near infrared
UV-Vis: Ultraviolet-visible
AR: Analytical purity
DMSO: Dimethyl sulfoxide
EDC: 1-(3-Dimethylamino propyl)-3-ethyl-carbodiimide hydrochloride
NHS: N-Hydroxysuccinimide
DPBF: 1,3-Diphenylisobenzofuran
CCK-8: Cell counting kit-8
DAPI: 4′,6-Diamidino-2-phenylindole, dihydrochloride
PBS: Phosphate-buffered saline
FBS: Fetal bovine serum
OD value: Optical density value.
